This article has been retracted.

# Neural Network Based on Health Monitoring Electrical Equipment Fault and Biomedical Diagnosis

**DOI:** 10.1155/2022/8358794

**Published:** 2022-08-21

**Authors:** Xinjun Zhang, Yingli Lyu

**Affiliations:** Department of Electrical Engineering, Jiyuan Vocational and Technical College, Jiyuan 459000, China

## Abstract

In order to improve the accuracy of electrical equipment failure diagnosis and keep electrical equipment operating safely and efficiently, this paper proposes to design an electrical equipment failure diagnosis system based on a neural network, analyze the faults of electrical equipment and their causes, and establish knowledge base according to relevant data and expert judgment. The fault knowledge base was introduced into the neural network operation structure, and the fault diagnosis results were classified step by step through multiple subnetworks. In data preprocessing, in order to avoid the redundancy of primary fault information features, the principal component heuristic attribute reduction algorithm was used to select the fault data samples optimally. The neural network learning algorithm is used to calculate the forward direction and error rate of the initial error data, and the reliability function is used to optimize the initial weight threshold of the neural network, propagating the error backwards and high. Experimental results show that adding attribute reduction improves error classification performance, avoids the problem of local minima through neural network operation, and has fewer iteration steps, lower average error, and higher accuracy of fault diagnosis, reaching 95.6%.

## 1. Introduction

In power system, electrical equipment is an important core to ensure power operation and transmission. In actual operation, the fault ratio of electrical equipment is high [1]. At present, the fault inspection and maintenance of electrical equipment mostly depend on the experience and judgment of the staff. It can no longer meet the operational requirements of modern energy systems [2]. Therefore, it is very important in practice to continue working on failure diagnosis technology for electrical equipment. In recent years, some scientists have been studying in this direction. Reference [3] proposes a framework for electrical equipment failure diagnosis systems based on MultiAgent technology. For monitoring individual electrical equipment, ODS is used to access Power Big Data which improves the access efficiency of Power Big Data. Management and control agent, analysis and diagnosis agent, and information-aware agent are used to realize the intelligentization of the fault diagnosis system. Under the environment of cooperative working mechanism, the specific tasks of agents are determined. The multiagent system is established to realize intelligent diagnosis of multiple electrical devices, but this method does not consider the fault diagnosis associated with multiple electrical devices, which has certain limitations. In reference [4], it is proposed to analyze the dissolved gas content in oil in electrical equipment by gas chromatograph to judge the hidden faults in electrical equipment. Taking a transformer as an example, the acetylene content in the oil chromatographic data of the pressure side oil tank exceeds the standard, and the opening inspection of the pressure side oil tank shows that the last screen lead-out line of the connecting flange is loose, resulting in discharge, which shows the effectiveness of the oil chromatographic data analysis method. However, this method is only suitable for the hidden faults in oil-filled electrical equipment, and its scope of application is limited. In reference [5], a hierarchical Bayesian fault diagnosis method based on kernel is proposed. The kernel method is introduced into the hierarchical Bayesian model, optimized by kernel principal component analysis, and a calculation model with simplified parameters is obtained by expectation maximization algorithm. Multiclass predictive diagnosis of circuit breaker faults is realized by combining fault tree, but the calculation process of this method is complex and the calculation redundancy is high. There are other inspection methods in Japan and abroad. B. Wavelet-based information filtering for fault diagnosis of electric propulsion systems on electric ships studies the faults of electric drives in electrical systems, filters rich information by using two-dimensional wavelet transform of sensor data, reduces the computational complexity of classifiers, and realizes fault diagnosis in electric drive sensors of electric ships [6]. There is also research on failure diagnosis based on electrical signature analysis for predictive maintenance of synchronous generators in large electrical systems. By applying the electrical characteristic analysis technology to the condition monitoring research of static var generator in large power system, the faults of stator electrical imbalance and mechanical dislocation are detected, and the electrical characteristics of wound rotor static synchronous generator are also discussed, including signal analysis suggestions, how to identify rotor faults according to fault modes, and the characteristics of bipolar static synchronous generator [7]. In addition, the traditional methods mentioned above are not standardized in obtaining fault data, and it is difficult to obtain useful information. Moreover, they rely on a comprehensive case base and expert experience, which brings great difficulties for accurate fault diagnosis.

Electrical equipment has complex structure and various fault modes, and the core of its diagnosis is fault classification [8]. The structure of neural network is simple, which is suitable for solving the problem of complex internal mechanism. It can approach any nonlinear function with arbitrary precision and adjust the threshold of network weights repeatedly through reverse learning, so as to minimize the difference between actual and expected output. Therefore, this paper proposes to design electrical equipment fault diagnosis system based on neural network. By consulting relevant literature and expert research data, the knowledge base of historical fault information diagnosis of electrical equipment is constructed to provide data support for the fault diagnosis system. The neural network architecture of electrical equipment fault diagnosis is constructed [9]. In order to improve the speed of fault diagnosis and classification, fault data are processed by multiple subneural networks, and data are transmitted in parallel and fused. In the neural network operation, the heuristic reduction algorithm of attribute principal component is used to construct the component function of attribute on the basis of difference matrix, which simplifies the original sample set and improves the training efficiency. Forward and error calculations of error data are performed by neural network. Based on this, the confidence function is used to optimize the initial weights and thresholds of the neural network, and the optimized results are captured and trained in the neural network. This provides reverse error transmission. It not only gives full play to the mapping ability of neural network generalization but also avoids the local minimum problem and improves the diagnosis accuracy. The effectiveness of this method in fault diagnosis of electrical equipment is verified by experiments.

## 2. Electrical Equipment Fault Diagnosis Knowledge Base Construction

The operation of electrical equipment needs the cooperation of various electrical components, and the fault is usually caused by the loss of control of electric energy or control information in the process of transmission, distribution, and conversion [10]. Common faults of electrical equipment include open circuit, short circuit, abnormal grounding, electric leakage, damage of electrical components, output error of electronic equipment due to electromagnetic interference, and accidental failure of control system components [11]. Electrical equipment failure may lead to extensive loss of personnel and property. Therefore, it is of great significance for fault diagnosis to collect the phenomena and causes of electrical equipment faults with high probability. The electrical equipment fault diagnosis knowledge base is constructed, and the electrical equipment fault characterization and fault causes are collected which includes basic facts, rules, and other relevant information [12, 13]. The information in the knowledge base comes from consulting a large number of literature studies and many domain experts, which is the key to determine the inference ability of the system. Some diagnostic knowledge is shown in Table 1.

In the system, the expression form of knowledge base is production rules, each rule corresponds to a conclusion, and the premises are represented by “AND”. For example, IF winding is overheated AND fuse is blown, THEN coil is heated.

## 3. Design of Fault Diagnosis Structure of Electrical Equipment Based on Neural Network

Neural network is a mathematical model derived from the human nervous system, which is an algorithm model for distributed parallel information processing [14]. This model processes information through a large number of neurons with nonlinear mapping ability. In the network, neurons are organized in the form of hierarchical structure [15–18], and the processing units on each layer are connected with neurons on other layers in a weighted way. Using error back propagation, a three-layer forward neural network model is obtained, with the specific structure as shown in Figure 1.

By studying many typical fault samples in the knowledge base, we can recall the flaws' associated characteristics. When a case is entered, the neural network will use associative memory to find the closest fault and then realize fault diagnosis. However, when diagnosing multiple fault modes, the neural network will have too many nodes, resulting in huge structure, redundant information, and slow processing speed [19]. Therefore, this paper designs and uses several subneural networks to diagnose faults from different sides, and then fuses the diagnosis results of the subnetworks, thus reducing the uncertainty of fault diagnosis and improving the recognition rate.

The neural network for fault diagnosis of electrical equipment designed in this paper is composed of three layers of networks connected in series [20, 21], which has the characteristics of fast data transmission rate in series structure. The specific structure is shown in Figure 2. In layer 2, each subnetwork is connected in parallel so as to avoid the phenomenon that information is not transmitted if a certain network fails in the series structure.

The fault diagnosis steps of electrical equipment mainly include following[22–24]:

1. collecting fault information and converting it into an input mode of a neural network
2. associating the fault knowledge base and outputting information classification results through forward calculation in each subneural network
3. The classification results are transmitted to the decision fusion network, and the accurate fault diagnosis results are obtained by global fusion calculation

## 4. Fault Diagnosis Algorithm of Electrical Equipment Based on Neural Network

### 4.1. Data Preprocessing

The electrical equipment fault data samples collected by each sensor are transmitted to the neural network, and after being associated with the fault knowledge base [25, 26].

Because of the redundancy between data, the spatial vector model is established by selecting feature words, and the original data are processed by the heuristic attribute reduction algorithm of principal components [27, 28], and the optimal selection is made to complete the data preprocessing. First, we need to extract fault feature words from fault statements, and the calculation formula is as follows:

(1) $$\begin{array}{c} A=\frac{h\sum_{i=1}^{n}x_{i}t}{\delta }. \end{array}$$

In the formula, *A* represents fault feature words, *h* represents fault feature word space vector, *t* represents correlation degree with fault knowledge base, *δ* represents fault feature word selection operator, and *x*_*i*_(*i*=1,2,…, *n*) represents fitness at the *i* fault data acquisition node. Chi-square test theory is used to select features, which can effectively measure the correlation between feature items and categories. The calculation formula is as follows:

(2) $$\begin{array}{c} B=\frac{{\left|t-p\right|}^{\alpha }}{I-A\text{cot}a}. \end{array}$$

In the formula, *p* represents the fault probability of electrical equipment, *α* is the fitness population, *I* is the imaginary number of the fault itemset in the corresponding fault knowledge base, and *a* is the constant.

Through the word frequency-inverse file frequency, the corresponding weight is calculated based on the selected characteristic frequency [25], and the conversion from words to vector space is completed. The calculation formula is as follows:

(3) $$\begin{array}{c} C=T\sqrt{\frac{B-I\text{cot}a}{\pi p^{2}}}. \end{array}$$

In the formula, *T* represents the frequency of fault feature words in the text.

In this way, the primary selection of electrical equipment fault characteristics is completed. But at this time, redundancy and compatibility exist among fault features, which will make the calculation of neural network complicated [26]. The principal component heuristic attribute reduction algorithm is used for reduction. The attribute weights of initial features are discretized by clustering. The number of clusters is *l*, and the calculation formula is as follows:

(4) $$\begin{array}{c} D=\sum_{i=1}^{n}pw_{i}+\frac{c\sqrt{d}}{Cl}. \end{array}$$

In the formula, *w*_*i*_ represents the component function of a certain attribute, *c* is the conditional attribute, and *d* is the decision attribute.

Through the principal component heuristic algorithm, the component values of each attribute are calculated by using the difference matrix, and the reduced fault characteristics are obtained. The calculation formula is as follows:

(5) $$\begin{array}{c} E=D\left\{\frac{\left[\sqrt{f}-X\right]}{{\left[cf+d\right]}^{2}}\right\}. \end{array}$$

In the formula, *X*=(*u*_*ij*_) represents the difference matrix, *u*_*ij*_ represents the elements of the *i* row and *j* column in the difference matrix, and *f* represents the specific value of the fault data on the conditional attribute.

After reduction, the features of fault decision are greatly reduced, the number of input nodes of neural network is reduced, the structure of neural network is simplified, the redundancy between fault data is removed, and the operation cost is reduced.

### 4.2. Subneural Network Learning Operation

The number of neurons in the input layer, hidden layer, and output layer is *L*, *M*, and *N*. *y*_*LM*_ and *y*_*MN*_ are the thresholds for the input and hidden layers, and the hidden and output layers, respectively. The activation functions of hidden layer and output layer are *g*(*m*) and *g*(*n*), respectively. *β* and *γ* represent the input and output of neurons, respectively. The sample set of fault data is *s*_*k*_=(*s*_1_, *s*_2_,…, *s*_*k*_), *k*=1,2,…, *L*. The expected output is *d*_*k*_=(*d*_1_, *d*_2_,…, *d*_*k*_), *k*=1,2,…, *N*. The hidden layer output is as follows:

(6) $$\begin{array}{c} \gamma_{M}=Eg\left(m\right)\sum_{k=1}^{L}s_{k}+\sum y_{LM}. \end{array}$$

The output of the network is as follows:

(7) $$\begin{array}{c} \gamma_{N}=Eg\left(n\right)\sum_{k=1}^{N}d_{k}+\sum y_{MN}. \end{array}$$

The forward calculation of the subneural network is finished at this point.

The second neuron's output error in the output layer is as follows:

(8) $$\begin{array}{c} o_{k}=d_{k}-\left(\gamma_{M}-\gamma_{N}\right). \end{array}$$

The sum of error energies of all neurons in the output layer is as follows:

(9) $$\begin{array}{c} W=\frac{1}{N}\sum_{k=1}^{N}o_{k}^{2}. \end{array}$$

The reliability function is introduced into the subneural network structure to identify the possible faults in electrical equipment and the reliability of fault judgment according to certain judgment rules [27]. According to the output error obtained above, adjust the subneural network's weight threshold. The following formula is used to calculate the weighting factor between the output layer and the concealed layer:

(10) $$\begin{array}{c} K={\left|W\right|}^{2}-\frac{2}{\theta }. \end{array}$$

In the formula, *θ* indicates credibility.

The adjusted weight threshold is transferred back to the input layer, and the weight coefficient between the input layer and the hidden layer is adjusted as follows:

(11) $$\begin{array}{c} Q=\left(\eta +\phi \right)K. \end{array}$$

In the formula, *η* represents the numerical gain coefficient and *ϕ* represents the inertia coefficient. The learning convergence speed is adjusted by these two coefficients, which are usually between [0,1]. The fault feature of the subneural network is recalculated, and the reverse transmission of error is realized.

### 4.3. Neural Network Decision Fusion

After completing the fault feature output of the subneural network, the feature vectors are fused, combined with random disturbance vector *φ*(*k*)=(*φ*_1_(*k*),*φ*_2_(*k*),*φ*_*i*_(*k*))^*T*^, after normalization, and the calculation formula is as follows:

(12) $$\begin{array}{c} R=o_{N}\varphi_{k}\text{cos}\left(\frac{2\pi }{W}\right){\left(\gamma_{M}+\gamma_{N}\right)}^{2}. \end{array}$$

By adding random disturbance value, enlarging the weight adjustment amount, speeding up the training speed of the network, and avoiding the parameter adjustment from entering the saturation state when the network parameters enter the saturation region, the neural network will jump out of the local minimum when fusing, ensuring that the network parameter adjustment will continue to keep the overall error convergence direction and complete the design of the failure diagnosis system for electrical equipment based on neural networks.

## 5. Experimental Results and Analysis

To test the application performance of the developed neural network-based electrical equipment malfunction diagnosis system, simulation experiments are needed. The neural network is trained by MATLAB simulation platform, the training function is trainlm, the learning rate is 0.1, the target error is 10^−5^, and the maximum number of iterations is 1000. The number of initial failure populations is 40, the selection parameter is 0.08, the crossover operator is 0.75, and the mutation probability is 0.01. Six kinds of fault voltage samples output by an electrical equipment are selected as test samples, and the reliability of fault diagnosis is tested by this method. The results are shown in Table 2.

It can be seen from the table that the reliability of this method in the fault diagnosis output of electrical equipment is higher, always above 0.97, which shows that the fault diagnosed is effective. The method of distributed electrical equipment fault diagnosis system based on multiagent technology in document [3], the application research method of oil chromatography analysis in oil-filled electrical equipment fault diagnosis in document [4], and the method of hierarchical Bayesian circuit breaker fault diagnosis based on kernel in document [5] is compared with the method in this paper. To comprehensively evaluate the performance of your design method, the number of convergence steps, the average absolute error of test samples, the maximum absolute error of test samples, and the accuracy rate are used to judge. The training error is shown in Figure 3.

From the figure, we can see that the method in this paper converged after 24 iterations, while the convergence iteration times of the methods in reference [3], reference [4], and reference [5] are 42, 65, and 80, respectively. By analyzing Figure 3, it can be seen that the method in this paper has reduced the error quickly with fewer iterations, while the error reduction rate of other methods is slow and fluctuates greatly. This is because this method preprocesses the fault data by using the heuristic reduction algorithm of attribute principal component, which greatly reduces the redundancy of calculation and can get the fault data processing result by using fewer iterations. The average absolute error, maximum absolute error, and accuracy of test samples are shown in Table 3.

After adding attribute reduction algorithm, the average absolute error is 4.73%, the accuracy rate is 95.6%, the average absolute error is 6.84%, the accuracy rate is 88.6%, the average absolute error is 8.4%, the accuracy rate is 90.5%, and the average absolute error is 10.35%. The accuracy of this method is far superior to other methods, and both the average absolute error and the maximum absolute error are far less than other methods, which show that the attribute reduction algorithm weakens the compatibility between fault data and is effective in classifying the original data.

In order to verify the anti-interference performance of the system designed in this paper, under different interference signal-to-noise ratios, the fault diagnosis speed of this method is compared with that of literature [3], literature [4], and literature [5], and the comparison results are shown in Table 4.

According to Table 4, when the interference signal-to-noise ratio is 48 dB, the fault diagnosis rate of this method is the longest, which is 5.86 ms, and the shortest, which is 4.32 ms, when the interference signal-to-noise ratio is 56 dB. The method in reference [3] has the longest fault diagnosis rate of 34.75 ms and the lowest rate of 28.34 ms under the interference signal-to-noise ratio of 56 dB. The method in reference [4] has the longest fault diagnosis rate of 29.35 ms and the lowest rate of 24.94 ms under the interference signal-to-noise ratio of 79 dB. The method in reference [5] has the longest fault diagnosis rate of 22.47 ms and the lowest rate of 19.54 ms under the interference signal-to-noise ratio of 79 dB. Comparing the fault diagnosis time of the four methods, it can be seen that the electrical equipment fault diagnosis rate of this method is the highest and the diagnosis efficiency is the best, which shows that the electrical equipment fault diagnosis system based on the neural network designed in this paper has better performance and can realize the electrical equipment fault diagnosis effectively and accurately.

## 6. Conclusion

With the continuous development of industrial enterprises, electrical equipment has been widely used. However, due to its frequent failures and diversified causes, its diagnosis has become a difficult point. In order to diagnose faults in electrical equipment efficiently and accurately, this paper proposes to design a fault detection system for electrical equipment based on neural network. Based on the establishment of electrical equipment fault knowledge base, several subneural networks are used to transfer the fault data so as to reduce the operation time and improve the efficiency of fault diagnosis. The attribute reduction algorithm is used to preprocess the fault data, eliminate the redundant information in the fault data, reduce the dimension of the fault information, extract the main characteristic parameters, optimize the original fault data, and effectively improve the operation speed and fault classification ability. Considering the elimination of diagnostic errors and deviations, the reliability function is introduced to optimize the initial weights and thresholds of the neural network when the neural network is used for the forward calculation and error calculation of fault data, and the reverse transmission training of errors is carried out to avoid the problem of local minima. Experiments show that the fault diagnosis system of electrical equipment based on neural network designed in this paper can effectively diagnose faults, with high reliability, less iteration steps, low average error, and fault diagnosis accuracy of 95.6%, which can provide theoretical support for fault diagnosis of electrical equipment and lay a foundation for practical application.

## Figures and Tables

**Figure 1:** Structure diagram of neural network.

**Figure 2:** Structure diagram of neural network for fault diagnosis of electrical equipment.

**Figure 3:** Comparison results of neural network error curves.

**Table 1:** Knowledge base for fault diagnosis of electrical equipment.

Fault symptom	Cause of failure
The two-phase insulation resistance of the motor is too low, the insulation of the wire skin is damaged, the coil is hot, and the vibration sound of the unit is loud	Winding overheating, winding insulation breakdown, fuse burning, and improper stator offline
The insulation resistance between stator winding conductor and iron core is too low, and the motor is overheated	The end of insulation aging winding touches the end cover, the power supply voltage is three-phase asymmetric, the voltage is too high, and the stator winding is short-circuited
Active and reactive loads of the unit decrease	Transmitter misoperation and feedback sensor failure

**Table 2:** Reliability results of electrical equipment fault diagnosis.

State code	Fault sample	Credibility
1	Failure 1	0.99
2	Failure 2	0.98
3	Failure 3	0.98
4	Failure 4	0.97
5	Failure 5	0.98
6	Failure 6	0.98

**Table 3:** Comparison of experimental results.

Experimental methods	Average absolute error of test sample (%)	Maximum absolute error of test sample (%)	Accuracy (%)
Methods of this paper	4.73	9.24	95.6
Method in reference [3]	6.84	13.26	88.6
Method in reference [4]	8.4	16.38	90.5
Method in reference [5]	10.35	20.72	92.1

**Table 4:** Comparison of fault diagnosis rate.

Interference SNR/dB	Methods of this paper/ms	Method in reference [3]/ms	Method in reference [4]/ms	Method in reference [5]/ms
12	5.52	28.34	25.88	18.61
28	5.42	29.12	24.94	19.54
36	5.57	32.12	25.34	19.76
48	5.86	33.46	28.64	20.45
56	4.32	34.75	27.41	19.86
65	4.98	30.34	28.64	21.64
79	5.63	31.36	29.35	22.47

## Data Availability

Data used to support this study are available on request.
